RETRACTED

# AS-tDR-007872: A Novel tRNA-Derived Small RNA Acts an Important Role in Non-Small-Cell Lung Cancer

**DOI:** 10.1155/2022/3475955

**Published:** 2022-06-16

**Authors:** Hang Fan, Hongbing Liu, Yanling Lv, Yong Song

**Affiliations:** ^1^Department of Respiratory Medicine, Jinling Hospital, Medical School of Nanjing University, Nanjing, 210093, Jiangsu, China; ^2^Department of Respiratory Medicine, Jinling Hospital, Nanjing Medical University, Nanjing, 210093, Jiangsu, China

## Abstract

tRNA-derived small RNAs (also known as tsRNAs) are novel kinds of non-coding RNAs. Although tsRNAs are aberrantly expressed in different tumor types, there is scanty of research investigating their expression profiling and functions in pulmonary adenocarcinoma (PADC). We identified the expression of AS-tDR-007872 in 30 non-small-cell lung carcinoma (NSCLC) patients' carcinoma tissues and conducted biological function evaluation. We also test the expression levels of AS-tDR-007872 in plasma samples obtained from 35 healthy people and 79 NSCLC cases. The results identified downregulated AS-tDR-007872 in both cancer tissues and plasma samples versus adjacent normal counterparts (*p* < 0.05) and healthy controls (*p* < 0.001). The area under the curve of AS-tDR-007872 was identified by receiver operating characteristic curve analysis to be 0.756 (95% CI, 0.663-0.849; *p* < 0.001). Furthermore, overexpression of AS-tDR-007872 in vitro inhibited tumor cell proliferation, invasion, and migration and promoted apoptosis. The knockdown of AS-tDR-007872 showed the opposite results. Meanwhile, we found significantly downregulated BCL2L11 after overexpressing AS-tDR-007872. From the above, our research suggests that AS-tDR-007872 can be a tumor suppressor and a promising biomarker for diagnosing lung cancer.

## 1. Introduction

Lung carcinoma (LC) is still the most prevalent cancer diagnosed and the prime reason for global cancer-related death nowadays [1]. Accounting for 75-80% of all LC, non-small-cell lung carcinoma (also known as NSCLC) has two major subtypes: lung squamous cell carcinoma (LSCC) and pulmonary adenocarcinoma (PADC). PADC is the most common histological subtype of LC [2]. Since LC is usually found in late-stage and is related to very poor 5-year overall survival [3], finding early and accurate diagnosis is important. Noninvasion detection of LC is currently based on computed tomography (CT) or other imaging techniques and the detection of serum tumor markers [4]. However, image exams usually lead to high false-positive rate [5], and serum tumor markers are limited by low sensitivity and specificity [6]. Therefore, the development of noninvasive biomarkers that could be used for early detection and prognosis of LC is still necessary. On the other side, tumor's sustained proliferation and metastatic potential lead to high mortality [7], so understanding molecular mechanisms underlying carcinoma cell apoptosis and multiplication is necessary [8, 9]. The critical role of some protein-coding gene (KRAS, TP53, and EGFR) mutations in the pathogenesis of NSCLC has been well established by multiple molecular epidemiological studies [10, 11]. Recent progress indicates that noncoding genes have become an indispensable role in the cancer paradigm [12].

RETRACTED

Noncoding RNAs can be categorized as either small or long ncRNAs according to their size, among which the former is vital in the modulation of gene expressions, such as miRNA and piRNA [13]. tsRNAs, consisting of tRNA halves (tiRNAs) and tRNA-derived RNA fragments (tRFs), belong to a novel kind of small ncRNAs that are reported to be linked to tumor formation, invasion, and metastasis [13]. It was initially described as a mechanism against phage infection in E. coli. Mature tRNAs are cleaved by angiogenin, a stress-activated ribonuclease in an anticodon loop, producing 5′ tiRNAs and 3′ tiRNAs [14]. Via replacing the eukaryotic initiation factor from the mRNA's m7G cap, natural or synthetic 5′ tiRNA transfection can suppress protein translation in bone cancer cells. These initiators are crucial to the 5′-UTR secondary structure conformation of the mRNA. Under the condition of cell stress, when the mature tRNA is specifically cleaved by angiopoietin, it will produce tiRNA, which is considered to be a transducer or effector involved in cell stress response. tiRNAs mainly promote the response of cells to stress by reprogramming translation, inhibiting apoptosis, degrading mRNA, and producing stress particles [15]. It has been reported that stress-induced tiRNAs can modulate the stress response [16], giving rise to stress granule assembly and protein synthesis inhibition. tRFs are another kind of tsRNAs obtained by precise processing of the 5′ or 3′ end of mature or precursor tRNAs and can be classified as either tRF-5, tRF-3, or tRF-1 series. tRFs can affect a wide spectrum of cell functions like multiplication and RNA inactivation through the cooperation of Argonaute. Reportedly, some tsRNAs promote the development of cancer [17].

Multiple evidences suggest that functional small RNAs have a dual role in carcinogenesis and tumor suppression. tsRNA is considered a promising potential biomarker for different types of tumors. To date, tsRNAs are reported to be related to B-cell lymphoma, breast cancer, liver cancer, and LC [18–20]. Increasing tsRNAs have been identified as potential biomarkers for cancer. For example, tRF-1001 is upregulated in many cancer cell strains of different lineages, suggesting its potential correlation with cell multiplication.

RETRACTED

Although tsRNA was discovered in the early 1990s [21], it was considered to be useless RNA and did not attract attention then. As novel RNAs, There are far too few studies of tsRNA in NSCLC. For the first time, we report that AS-tDR-007872 is associated with LC. We first discovered low AS-tDR-007872 expression in both LC tissues and plasma. We found tRNA-5 is one with the richest expression in both LC tissues and normal counterparts, which is consistent to other researches. However, further research about the biological mechanism of AS-tDR-007872 in lung cancer has not been studied. Thus, the motivation and purpose of this study is to investigate whether AS-tDR-007872 regulated lung cancer development and discuss its functional mechanisms so as to provide novel insights into lung cancer treatment.

## 2. Data and Methods

### 2.1. Patients and Specimens

The specimens were paired NSCLC samples and adjacent normal counterparts obtained from 30 patients with NSCLC surgery in Thoracic Surgery, Jinling Hospital, Medical School of Nanjing University between November 2011 and September 2012.  Table 1 summarizes clinicopathological characteristics of NSCLC patients. Once the tissue samples were surgically removed, they were subjected to liquid nitrogen freezing (-80°C) for storage until RNA was extracted. We collected plasma from 35 healthy people and 79 newly diagnosed LC cases in the Jinling Hospital in Nanjing, China between January 2018 and January 2019. Tumor patients are classified according to TNM malignant tumors. The study has obtained the approval from the Institutional Review Board of Nanjing University, with informed consent obtained from each participant.  Table 2 shows NSCLC patients' clinicopathological data. Sample processing was performed within 2 hours after collection. After complete separation of blood cells by centrifugation (1200 g, 4°C, 10 minutes), the supernatant plasma was gathered carefully and the specimens were stored at 80°C until further analysis.

### 2.2. Cell Cultivation

We purchased 7 NSCLC cell strains (HBE, A549, HCC827, PC-9, H-1299, H-1975, and SPCA1) from Institute of Biochemistry and Cell Biology, Chinese Academy of Sciences (Shanghai, China). Of them, A549, HCC827, H-1299, HBE, and H-1975 were immersed in RPMI 1640 minimal medium (GIBCO-BRL; Invitrogen, Carlsbad, CA) for cultivation, while the other two in DMEM (GIBCO-BRL; Invitrogen). Then, into the basic culture medium + 100 units/mL penicillin + 100 *μ*g/mL streptomycin, thermal inactivated 10% fetal calf serum (FBS) and antibiotics were placed, and cell cultivation was conducted in a humidified incubator under the conditions of 37°C and 5% CO_2_.

RETRACTED

### 2.3. RNA Separation and qRT-PCR Analysis

TRIZOL reagent (Invitrogen) isolation of total RNA from refrigerated tissue or treated cells was carried out by referring to the supplier's recommendations. For AS-tDR-007872 determination, miRNA First Strand cDNA Synthesis (Tailing Reaction) (Sangon Biotech, China) was used to reverse transcribe the isolated RNA into cDNA. Then, AS-tDR-007872 quantification was performed following the supplier's recommendations with the use of SYBR Premix Ex Taq II (Perfect Real Time; TaKaRa). The following is the gene-specific primers: GAPDH sense (5′-3′) GTCAACGGATTTGGTCTGTATT, anti-sense (5′-3′) AGTCTTCTGGGTGGCAGTGAT; BCL2L11 sense (5′-3′) AAGGTAATCCTGAAGGCAATCA, anti-sense (5′-3′) CTCATAAAGATGAAAAGCGGGG, AS-tDR-007872 (5′-3′) GCCAGGGATTGTGGGTTCGA. GAPDH was utilized for standardization. With the use of the ABI7500 real-time PCR system supplied by Applied Biosystems, Foster City, CA, a PCR reaction was performed at 95°C for 30 s and then a cycle of 40 s at 95°C for 5 s and a cycle of 34 s at 60°C. qRT-PCR was run in triplicate. Cytoplasmic and nuclear RNA were separated and purified via the MagMAX™ mirVana™ Total RNA Isolation Kit (Thermo Fisher Scientific, New Hampshire, USA) by referring to the supplier's recommendations. The relative expression quantification of AS-tDR-007872 with reference to GAPDH was calculated via the 2^-△△CT^ formula. qRT-PCR product was identified as AS-tDR-007872 sequence by sanger sequencing.

### 2.4. Transfection

Mimics and inhibitor (Ribo Life Science Co.) transfections into cells were conducted by referring to the supplier's recommendations of Lipofectamine 2000 (Invitrogen, Shanghai, China). Chaotic RNA sequences of the same sequence length were used for standardization. Cells were used for further experiments after 24 h transfection.

### 2.5. Cell Multiplication and Colony Formation Assays

The monitoring of cell multiplication used Cell Proliferation Kit I (MTT; Roche Applied Science). A549 and SPCA1 after AS-tDR-007872 mimics or control mimics transfection were placed in the wells of 96-well plates. Cell multiplication was recorded at a frequency of 24 hours. For cell colony formation, 300 A549 and SPCA1 cells transfected with AS-tDR-007872 or control mimics were placed in new 6-well plates that were kept in a 10% FBS-containing medium and renewed 4 days per time. One week later, the colonies formed were subjected to methanol immobilization and crystal violet staining (0.1%; Sigma-Aldrich, St. Louis, MO). The clones were counted by Image-Pro Plus (Version 6.0, Media Cybernetics). H1299 and H1975 cells were treated with AS-tDR-007872 inhibitors or control inhibitor transfection.

RETRACTED

### 2.6. Transwell Assay

Transwell analysis was performed with a polycarbonate Transwell filter (Corning CostarCorp, Cambridge, MA). The bottom chamber filled with 10% FBS-filled medium. Cells (5∗10^4^) after 24 h of treatment with AS-tDR-007872 mimics or control mimics were processed for suspension in the culture medium and seeding into the apical chamber. Following culturing at 37° C for 24 hours, those staying on the lower surface were subjected to paraformaldehyde immobilization and crystal violet dyeing (0.1%; Sigma-Aldrich). The number of invading cells was observed under the optical microscope (Leica, Germany) and was counted by Image-Pro Plus.

### 2.7. Apoptosis and Cell Cycle by Flow Cytometry

Cells with AS-tDR-007872 or control mimics transfection were cultivated in the wells of 6-well plates for 24 hours and harvested by trypsinization. Cells were harvested post FITC-annexin V propidium iodide (PI) dual staining, followed by analysis via flow cytometry (FCM) (FACScan) and CellQuest both supplied by BD Biosciences, USA. For FCM, a Cycle TEST™ PLUS DNA Kit (BD Biosciences) was used. PI staining of cells was then performed by referring to the protocol and analyzed by FACS tank, for the calculation and comparison of the percentage of S-, G0/G1-, and G2/M-phase cells.

### 2.8. Western Blotting

SPCA1 and A549 cells after AS-tDR-007872 or control mimics transfection were treated with a lysis buffer comprising mammalian protein extraction reagent RIPA (Beyotime, China)+PMSF (Roche) + protease inhibitor mix (Roche, Basel, Switzerland). Then, a Bio-Rad protein assay kit measured the protein concentration. Thereafter, specimens comprising 50 mL protein were run on a 15% SDS-PAGE before transferring to a 0.22 mm nitrocellulose membrane (Sigma-Aldrich) and cultivation with specific antibodies. ECL detected specific bands, and Densitometry using Quantity One Software (Bio-Rad, Hercules, California) was conducted for protein expression analysis. GAPDH served as a control. Anti-BCL2L11 antibody and Anti-GAPDH antibody were supplied by Abcam (# ab32158) and Sigma-Aldrich (USA), respectively.

### 2.9. Statistical Processing

All statistical analyses used SPSS 23.0 (IBM, Chicago, USA), with *p* < 0.05 as the significance level. Categorical data were given as *n*(%), and a chi-squared test was applied. Measurement data were given as the mean ± SD, and the difference was analyzed using the two-tailed Student's *t*-test. Mann–Whitney*U*test, Kolmogorov-Smirnov*Z*test, and Moses and Wald-Wolfowitz test were applied for the comparison of the expression levels of plasma AS-tDR-007872 in NSCLC patients and healthy controls.

RETRACTED

## 3. Results

### 3.1. AS-tDR-007872 Was Decreased in the LC Tissue Samples versus Their Adjacent Counterparts

We prepared 3 high-quality paired PADC and adjacent normal tissue samples for high-throughput sequencing. tsRNAs were found to present different expression profiles between PADC and adjacent normal tissues (Supplementary material Figures 1 and 2). Because of low levels of tsRNAs generated from precursor tRNAs, we focused on mature tsRNAs that can be further categorized as either tRNA-5 (5-terminal of mature tRNA, 5′ tRH and 5′ tRF), itRF (internal of mature tRNA, tRF-i) or tRNA-3 (3-terminal of mature tRNA, 3′ tRH and 3′ tRF)∗∗ based on their location. As shown in supplementary material Figure 2, tRNA-5 is the one with the most abundant expression in both LC tissues and adjacent counterparts.

High-throughput sequencing and bioinformatics analysis identified 11 high-expression tsRNAs and 25 low-expression tsRNAs (Supplementary material Figure 1B). qRT-PCR was then performed on 30 matched clinical NSCLC tissues and adjacent counterparts to determine whether these tsRNAs were differentially expressed in the disease. We found statistically downregulated AS-tDR-007872 in clinical NSCLC samples versus adjacent counterparts (*p* < 0.05; Figure 1). Besides, evaluation of the association of AS-tDR-007872 with clinical pathology parameters was carried out (Table 1). The results showed that age, gender, differentiation, or stage was not related to the expression of AS-tDR-007872 (*p* > 0.05).

### 3.2. Plasma AS-tDR-007872 Was Downregulated in LC Patients versus Healthy Volunteers

To examine the diagnostic potential of AS-tDR-007872, 114 plasma specimens comprising 79 NSCLC samples and 35 non-NSCLC samples, were analyzed. There is no data loss during detection. The study revealed downregulated plasma AS-tDR-007872 in LC patients versus normal controls (Figure 2(a)). Real-time PCR was then performed on these specimens for further analysis, and the*p*values of Mann–Whitney*U*test, Kolmogorov-Smirnov*Z*test, and Moses and Wald-Wolfowitz test were below 0.05.

Subsequently, the correlation of AS-tDR-007872 with various NSCLC clinical characteristics was examined. As is shown in Figures 2(b) and 2(c), the expressions of AS-tDR-007872 were linked to smoking (*p* < 0.001) and the pack-years of patients. Meanwhile, no evident association was determined between plasma AS-tDR-007872 of NSCLC patients and their gender, age, tumor size, lymphatic metastasis, or histology type.

The evaluation of the predictive efficacy of AS-tDR-007872 employed ROC curve analysis. The area under the ROC curve (AUC) was 0.756 (95% CI, 0.663-0.849; *p* < 0.001), with the optimal sensitivity being 0.857 and specificity being 0.519 for distinguishing NSCLC cases from healthy controls. On this basis, we further evaluated the value of AS-tDR-007872 in distinguishing NSCLC patients of different stages. As indicated by ROC analyses, the AUCs of AS-tDR-007872 in distinguishing stage I-II, stage III, and stage IV patients from controls were 0.706 (95% CI 0.531–0.881), 0.779 (95% CI 0.657–0.900), and 0.772 (95% CI 0.672–0.873), respectively.

RETRACTED

### 3.3. Overexpression of AS-tDR-007872 Reduced Proliferation in NSCLC Cell Lines

Using qRT-PCR, we measured AS-tDR-007872 expression in NSCLC cell stains, so as to understand its role in NSCLC development. AS-tDR-007872 expression was comparatively underexpressed in 5 LC cell lines A549, H-1299, PC-9, H-1975, and SPCA1 versus HBE cells, whereas slightly elevated AS-tDR-007872 was observed in H-1975 compared with HBE cells (Figure 3(a)). Considering the lowly expressed AS-tDR-007872, we used AS-tDR-007872 mimics to over-express in A549 and SPCA1 cell lines and over 100 times higher expression of AS-tDR-007872 than the control was confirmed by qRT-PCR (Supplementary material Figure 3). Meanwhile, we used the AS-tDR-007872 inhibitors to decrease the expression of AS-tDR-007872 in H-1299 and H-1975 cell strains.

In comparison with control cells, AS-tDR-007872 mimics transfection led to evidently reduced A549 and SPCA1 cell viability as indicated by the MTT assay results (Figure 3(c)). Also, the colony formation assay results showed notably weakened colony formation capacity of the population by overexpressing AS-tDR-007872 (Figure 3(b)). Additionally, transfection with AS-tDR-007872 knockdown inhibitors in H-1299 and H-1975 revealed a corresponding increase comparing to control groups in MTT as well as colony formation assays.

### 3.4. Overexpression of AS-tDR-007872 Suppressed NSCLC Cell Migration and Invasiveness

There is no study elucidating the impact of AS-tDR-007872 on NSCLC cell migration and invasiveness. Hence, we further used the transwell assay for confirmation. AS-tDR-007872 overexpression decreased cell migration, as well as invasion in A549 and SPCA1. Instead, cells transfecting AS-tDR-007872 knockdown inhibitors promoted migration and invasion (Figures 4(a) and 4(b)).

### 3.5. Overexpression of AS-tDR-007872 Promoted Apoptosis but Had No Effect on Cell Cycle in NSCLC Cell Lines

Apoptosis as a major mechanism for programmed cell death; its defects can drive genomic instability and tumorigenesis. To investigate the involvement of AS-tDR-007872 in modulating NSCLC cell apoptosis, A549 and SPCA1 were transfected, respectively, with AS-tDR-007872 mimics and control mimics. Cells were harvested 48 h after transfection for FCM analysis. AS-tDR-007872 overexpression significantly promoted apoptosis, whereas H-1299 cells transfected with inhibitors of AS-tDR-007872 showed reduced apoptosis (Figure 4(c)). It suggests a critical role of AS-tDR-007872 in LC cell apoptosis.

RETRACTED

No studies have demonstrated the effect of AS-tDR-007872 on the cell cycle of NSCLC cell strains. As shown in Supplementary material Figure 4, the experimental results indicate that overexpression of AS-tDR-007872 does not affect the cell cycle of NSCLC cell lines.

### 3.6. BCL2L11 Had Low Expression in AS-tDR-007872 Mimics-Transfected A549 and SPCA1

Considering tsRNAs have similar structures with miRNAs to some extent, the downstream target genes of AS-tDR-007872 was forecast with the TargetScan (URL: http://www.targetscan.org/), which returned 144 genes (Supplementary material Figure 5A). Then, we use KEGG (https://www.kegg.com/) to analyze these 144 genes. The results showed that 11 genes were related to cancer in this list, including BCL2L11, JAG1, FGFR1, IFNGR2, IGF1, IKBKB, JAK1, KIT, STK4, WNT5A, and CALM3 (Supplementary material Figure 5B). We detected with real-time PCR the expressions of these 11 genes in AS-tDR-007872 mimics-transfected A549 and SPCA1. We found that except for BCL2L11 and CALM3 (Figures 5(a) and 5(b)), which have consistently low expression in A549 and SPCA1; the expressions of the other 9 genes in these two cell lines were not consistent. This result indicates that BCL2L11 and CALM3 may be downstream target genes of AS-tDR-007872.

### 3.7. BCL2L11 Had High Expression in LC Tissues

We consulted the open database Oncomine (https://www.oncomine.org/) for the expression of BCL2L11 and CALM3 in LC (Supplementary material Figure 6). BCL2L11 was found to be overexpressed in LC (*p* = 0.008), while the expression of CALM3 was not different between NSCLC and normal people. Besides, we detected BCL2L11 in 30 paired NSCLC tissues and adjacent counterparts by real-time PCR and found highly expressed BCL2L11 in carcinoma tissues (Figure 5(c)).

### 3.8. Overexpressing AS-tDR-007872 Reduced the Expression of BCL2L11 in A549 and SPCA1

We detected BCL2L11 expression by real-time PCR in AS-tDR-007872 mimics-transfected A549 and SPCA1. As shown in Figure 5(a), overexpression of AS-tDR-007872 reduced BCL2L11 expression. Moreover, Western Blot detected BCL2L11 protein levels when overexpression or knockdown AS-tDR-007872 in LC cell strains. In A549 and SPCA1, overexpressing AS-tDR-007872 reduced BCL2L11 protein levels (Figure 5(d)), and knocking down AS-tDR-007872 increased BCL2L11 protein levels. That indicates that AS-tDR-007872 regulates apoptosis by reducing the expression of BCL2L11.

RETRACTED

## 4. Discussion

In the past, ncRNA was considered junk in evolution, but increasing evidence suggests that they have functional molecular mechanisms. Noncoding RNAs are classified as 2 subclasses according to a threshold of 200 nucleotides (nt). Small or short ncRNAs are under 200-nucleotide-long, and long noncoding RNAs (lncRNAs) are >200 nt, while microRNAs (miRNAs) with a size of ~20 nt are the most famous sncRNAs. miRNAs can negatively regulate gene expression and induce degradation or inhibit translation by binding to the target mRNA. There is growing evidence that miRNAs can be therapeutic targets or biomarkers for many diseases. tsRNAs was first described as a mechanism against phage infection in E. coli. But it did not get much attention at the time. With the advances in sequencing technology, the next generation sequencing technology in particular [22], tiRNA has been reidentified in different cells and tissues. In the last ten years, tRNA and tsRNAs have been shown to be dysregulated in cancer and are involved in the development of cancers like breast cancer [23], ovarian cancer [24], and colorectal cancer [25]. A research revealed upregulated TRF-Leu-CAG RNA in NSCLC tissues and cell lines [20] and the capacity of tRF-Leu-CAG to enhance cell multiplication, affect cell cycle, and regulate AURKA expression. Nicholas et al. identified four tRNA-derived small RNAs (tsRNA), ts-19, ts-29, ts-46, and ts-112, that exhibit significant alterations in expression profiles following RUNX1 deregulation in normal mammary epithelium and malignant breast tumor cell models [26]. Although tsRNAs has received widespread attention, the biological functions and molecular mechanisms of tsRNAs in NSCLC are still poorly understood. For the first time, our data indicate statistically downregulated AS-tDR-007872 in 5 of 6 LC cell strains compared with HBE and plasma. The experiment of gain function of AS-tDR-007872 in LC cells identified significantly suppresses cell multiplication, migration, and invasiveness by overexpressing AS-tDR-007872. Meanwhile, when knocking down AS-tDR-007872, LC cell lines showed enhanced multiplication, migration, and invasion. Moreover, gain-of-function and loss-of-function analysis results identified that AS-tDR-007872 expression is a necessary and sufficient condition for NSCLC cell apoptosis, which suggests the potential role of AS-tDR-007872 as an antioncogene in LC. Besides, we found tRNA-5 is the tsRNA with the richest expression in both LC tissues and adjacent counterparts, which is consistent to other researches.

RETRACTED

Many research shows that tRF is a miRNA-like fragment, works in a similar way through the Argonaut protein interaction, and is involved in the production of DICER^26^. However, we also found AS-tDR-007872 could regulate downstream target genes. Herein, we found the downstream target gene of AS-tDR-007872—BCL2L11 by bio database and bioinformatics analysis. By searching Oncomine, we found BCL2L11 was highly expressed in LC. When AS-tDR-007872 was upregulated in LC cell strains, BCL2L11 was suppressed at the protein, as well as the mRNA level. When we knock down AS-tDR-007872, the expression of BCL2L11 was increased.

Since tsRNAs have short nucleotide sequences and stable structures, tsRNAs considered to be promising potential biomarkers for different kinds of tumors. To date, there is no research quantifying AS-tDR-007872 transcript levels in plasma. This study is aimed at clarifying the diagnostic utility of plasma circulating AS-tDR-007872 in NSCLC. First, the diagnostic value of plasma AS-tDR-007872 in distinguishing NSCLC cases from controls was investigated. Using reverse transcription-qPCR to measure the expression levels of AS-tDR-007872, we demonstrated that AS-tDR-007872 was significantly deregulated in plasma samples of NSCLC patients, which correspond with the expression of AS-tDR-007872 in NSCLC tissues. We find that in NSCLC patients, AS-tDR-007872 was associated with smoking and the pack-years but not with sex, lymphatic metastasis, tumor size, or histology type, probably because of the correlation of tsRNAs with oxidative stress. Moreover, AS-tDR-007872 had an AUC of 0.779 (95% CI: 0.657–0.900) in distinguishing stage III and of 0.772 (95% CI: 0.672–0.873) in distinguishing stage IV patients from controls, which seem to be more sensitive than the AUC (95% CI: 0.531–0.881) of AS-tDR-007872 in distinguishing stage I-II patients from controls. AS-tDR-007872 appears to be a feasible biomarker for LC diagnosis.

Still, the current study shows some deficiencies. To begin with, the tumor sample size is small. Besides, the downstream mechanisms of AS-tDR-007872 are not covered. Thus, further research on related downstream genes and pathway mechanisms in a larger lung cancer sample size is needed to validate our conclusions.

## Figures and Tables

**Figure 1:** Relative AS-tDR-007872 expression in NSCLC tissues. (a, b) qRT-PCR analysis of AS-tDR-007872 expression relative to GAPDH in NSCLC tissues (*n* = 30) and normal counterparts (*n* = 30).

**Figure 2:** Expression levels of plasma AS-tDR-007872 in NSCLC patients and healthy controls. (a) AS-tDR-007872 was significantly down-regulated in NSCLC patients (*n* = 79) compared with healthy controls (*n* = 35). (b, c) Plasma AS-tDR-007872 expression levels in NSCLC were associated with smoking and the pack-years of patients. (d) The AUC of the ROC of AS-tDR-007872 for plasma of NSCLC patients equaled 0.756 (95% CI, 0.663–0.849; *p* < 0.001). AUC: area under the receiver operating characteristic (ROC) curve.

RETRACTED

**Figure 3:** AS-tDR-007872 reduced proliferation in NSCLC cell lines. (a) Expression levels of AS-tDR-007872 in NSCLC cell lines. (b) Proliferation of AS-tDR-007872 mimics or inhibitor-transfected cell lines by colony-forming assay. (c) Proliferation of AS-tDR-007872 mimics or inhibitor-transfected cell lines by MTT assay. The data (mean ± SD) were from experiments run independently for three times. ^∗^*p* < 0.05*vs.* HBE/Control/NC group.

**Figure 4:** The effect of AS-tDR-007872 on NSCLC cell migration, invasion, and apoptosis. (a, b) Representative images of Boyden chamber assay used to determine AS-tDR-007872's effects on cell migration and invasiveness. (c) AS-tDR-007872 promoted apoptosis in NSCLC cell lines. Flow cytometry analyzed the percentage of apoptotic cells. The data (mean ± SD) were from experiments run independently for three times. ^∗^*P* < 0.05*vs.* the Control group.

**Figure 5:** Expression levels of BCL2L11 in NSCLC cell lines and tumor tissues. (a, b) The expressions of BCL2L11 and CALM3 of A549 and SPCA1 transfecting with AS-tDR-007872 mimics. (c) Expression of BCL2L11 in 30 paired NSCLC tissues and adjacent counterparts by real-time PCR. (d) Expression of BCL2L11 was presented and evaluated in cells. The results were from experiments run independently for three times. GAPDH was the internal control. ^∗^*p* < 0.05*vs.* the Control group.

**Table 1:** Correlation of AS-tDR-007872 with clinicopathological characteristics of lung cancer.

Clinicopathological parameters	n	AS-tDR-007872 expression		
		Low	High	*p* value^a^
Age				0.542
≤65	23 (76.7)	16 (53.3)	7 (23.3)	
>65	7 (23.3)	4 (13.3)	3 (10.0)	
Sex				0.605
Male	14 (46.7)	10 (33.3)	4 (13.3)	
Female	16 (53.3)	10 (33.3)	6 (20.0)	
Differentiation				0.197
Moderate-well	27 (90.0)	19 (63.3)	8 (26.7)	
Poor	3 (10.0)	1 (3.3)	2 (6.7)	
Tumor size				0.083
≤5 cm	25 (83.3)	15 (50.0)	10 (33.3)	
>5 cm	5 (16.7)	5 (16.7)	0 (0)	
Primary location				0.605
Left lung	16 (53.3)	10 (33.3)	6 (20.0)	
Right lung	14 (46.7)	10 (33.3)	4 (13.3)	
Lymph node metastasis				1.000
Positive	12 (40.0)	8 (26.7)	4 (13.3)	
Negative	18 (60.0)	12 (40.0)	6 (20.0)	
TNM staging				0.301
I	14 (46.7)	8 (26.7)	6 (20.0)	
II/III/IV	16 (53.3)	12 (40.0)	4 (13.3)	
Smoke				0.429
Yes	12 (40.0)	9 (30.0)	3 (10.0)	
No	18 (60.0)	11 (36.7)	7 (23.3)	

^a^Chi-squared test.

RETRACTED

**Table 2:** Correlation between AS-tDR-007872 expression and clinicopathological parameters of lung cancer.

	NSCLC (%)	Healthy volunteers (%)	*p* value^a^
Gender			0.084
Male	54 (68.4)	18 (51.4)	
Female	25 (31.6)	17 (48.6)	
Age (years)			
≥65	38 (48.1)	3 (8.6)	
<65	41 (51.9)	32 (91.4)	
Histological subtype			
PADC	52 (65.8)		
LSCC	27 (34.2)		
Pathological tumor size			
T1/T2	25 (31.6)		
T3/T4	54 (68.4)		
Pathological lymph node metastasis			
Positive	60 (75.9)		
Negative	19 (24.1)		
Pathological stage			
I-IIIA	22 (27.8)		
IIIB-IV	57 (72.2)		
Smoking habit			
Yes	37 (46.8)		
No	42 (53.2)		
Pack-years			
0	37 (46.8)		
1-20	12 (15.2)		
21-49	16 (20.3)		
>49	14 (17.7)		

^a^Chi-squared test. NSCLC: non-small-cell lung carcinoma; PADC: pulmonary adenocarcinoma; LSCC: lung squamous cell carcinoma.

## Data Availability

The labeled dataset used to support the findings of this study is available from the corresponding author upon request.

## Supplementary Materials

Supplementary 1 Supplementary material Figure 1: high-throughput sequencing results of 3 paired lung adenocarcinoma and adjacent normal tissue samples. (A) tRNA derived small RNAs have different expression profiles between lung adenocarcinoma tissues and adjacent counterparts (Ad: lung adenocarcinoma tissue samples; dN: adjacent counterparts). (B) In combination with bioinformatics analysis, it showed 11 high-expression tsRNAs and 25 low-expression tsRNAs.

Supplementary 2 Supplementary material Figure 2: high-throughput sequencing results of 3 paired lung adenocarcinoma and adjacent normal tissue samples showed that different kinds of tsRNAs have different expressions but tiRNA-5 is the most abundant tsRNA in both lung adenocarcinoma tissues and adjacent normal tissues (AD: lung adenocarcinoma tissues, ADN: adjacent normal tissues).

Supplementary 3 Supplementary material Figure 3: transfection efficiency of AS-tDR-007872 mimics in A549 and SPCA1 cell lines by qRT-PCR technique.

Supplementary 4 Supplementary material Figure 4: AS-tDR-007872 had no effect on NSCLC cell cycle. Data are from experiments run independently for 3 times.

Supplementary 5 Supplementary material Figure 5: (A) the 144 downstream target genes of AS-tDR-007872 predicted by TargetScan. (B) The 11 genes related to cancer predicted by KEGG.

Supplementary 6 Supplementary material Figure 6: Oncomine showed the expression of BCL2L11 and CALM3 in lung cancer.
